# 3D Model of Lamprey Estrogen Receptor with Estradiol and 15α-Hydroxy-Estradiol

**DOI:** 10.1371/journal.pone.0006038

**Published:** 2009-06-25

**Authors:** Michael E. Baker, David J. Chang, Charlie Chandsawangbhuwana

**Affiliations:** 1 Department of Medicine, University of California San Diego, La Jolla, California, United States of America; 2 Department of Biology, University of California San Diego, La Jolla, California, United States of America; 3 Department of Bioengineering, University of California San Diego, La Jolla, California, United States of America; Tel Aviv University, Israel

## Abstract

**Background:**

Lamprey, basal vertebrate, is an important model system for understanding early events in vertebrate evolution. Lamprey contains orthologs of the estrogen receptor [ER], progesterone receptor and corticoid receptor. A perplexing property of lamprey is that 15α-hydroxy-steroids are active steroids. For example, 15α-hydroxy-estradiol [15α-OH-E2] is the estrogen, instead of estradiol [E2]. To investigate how 15α-OH-E2 binds lamprey ER, we constructed a 3D model of the lamprey ER with E2 and 15α-OH-E2.

**Methodology:**

We used the 3D structure of human ERα as a template to construct a 3D model of lamprey ER. E2 and 15α-OH-E2 were inserted into the 3D model of lamprey ER and 15α-OH-E2 was inserted into human ERα. Then the each steroid-protein complex was refined using Discover 3 from Insight II software. To determine if lamprey ER had some regions that were unique among vertebrate ERs, we used the ligand-binding domain of lamprey ER as a query for a BLAST search of GenBank.

**Principal Findings:**

Our 3D model of lamprey ER with 15α-OH-E2 shows that Sδ on Met-409 can form a hydrogen bond with the 15α-hydroxyl on 15α-OH-E2. In human ERα, the corresponding residue Ile-424 has a van der Waals contact with 15α-OH-E2. BLAST analysis of GenBank indicates that among vertebrate ERs, only lamprey ER contains a methionine at this position. Thus, the contact between Sδ on Met-409 and 15α-OH-E2 is unique. Interestingly, BLAST finds that five New World monkeys and a sturgeon contain a valine instead of isoleucine.

**Significance:**

In addition to shedding light on the structure of the ER in a basal vertebrate, our 3D model of lamprey ER should prove useful in virtual screening of chemical libraries to identify compounds for controlling reproduction in sea lamprey, an environmental pest in Lake Michigan.

## Introduction

Lamprey and hagfish are two primitive fish at the base the vertebrate line, which has motivated studies of these fish to understand early events in vertebrate evolution [1]–[3]. In particular, sea lamprey (*Petromyzon marinus*) is of interest for understanding the origins of adrenal and sex steroid signaling [4]–[10] because orthologs of vertebrate estrogen receptor [ER], progesterone receptor [PR] and a corticoid receptor [CR] have been cloned from sea lamprey [7]. A puzzle about sea lamprey is that the principal estrogens, androgens and progestins in its serum differ from that in humans [11]–[14]. For example, lamprey serum contains 15α-hydroxy-estradiol [15α-OH-E2] and 15α-hydroxy-estrone [15α-OH-E1] and low levels of estradiol [E2], which is the main estrogen in land vertebrates and bony fish [Figure 1]. Lamprey serum also contains 15α-OH-progesterone and 15α-OH-testosterone and low levels of progesterone and testosterone. These data suggest that 15α-hydroxy-steroids are the active steroids in lamprey.

**Figure 1:** Structures of estradiol and 15α-hydroxy-estradiol. Estradiol is the biologically active estrogen in most vertebrates. 15α-hydroxy-estradiol is found in lamprey blood [11], [12] and may be the biologically active estrogen.

To determine if there is a structural basis in lamprey ER for the recognition of 15α-OH-E2, we constructed a 3D model of lamprey ER complexed with E2 and 15α-OH-E2. This 3D model shows that Sδ on Met-409 in lamprey ER can have a hydrogen bond with 15α-hydroxyl on 15α-OH-E2. In human ERα, the corresponding residue is Ile-424, which has a van der Waals contact with 15α-OH-E2. A BLAST [15] search of GenBank found that almost all other vertebrate ERs contain an isoleucine and none contain a methionine at this position. The uniqueness of lamprey Met-409 and its stabilizing interaction with the 15α-hydroxyl on 15α-OH-E2 suggests that it may be possible to find chemicals that selectively inhibit lamprey ER by using our 3D model of lamprey ER as a template for virtual screening of chemical libraries. Such chemicals could be used to control reproduction of *P. marinus*, which is a pest in the Great Lakes in the USA.

### Experimental Construction of 3D Models

The 3D structure of human ERα [PDB: 1G50] was used as a template for constructing the 3D model of lamprey ER. The sequences of the steroid-binding domain of lamprey ER and human ERα are 57% identical without any gaps [Figure 2]. This strong similarity between lamprey ER and its template gives us confidence in the accuracy lamprey 3D model. We used the Multiple Mapping Method (MMM) software [16] to construct the 3D model of lamprey ER. We selected three alignment algorithms Muscle, Align2D and ClustalW to align the target sequence [lamprey ER] and the human ERα template [1G50]. MMM takes each alignment and constructs a composite alignment, which is then used by Modeller [17] to construct the 3D model of lamprey ER.

**Figure 2:** Alignment of lamprey ER with human ERα and human ERβ. α-helices and β-strands from the crystal structures of ERα and ERβ are shaded in each sequence and notated below the alignment. Residues in human ERα involved in binding of estradiol are shown in green. Glu-419, which stabilizes His-524 is shaded in brown. Crystal structure accessions are human ERα [PDB: 1G50], human ERβ [1QKM].

After we obtained the apo-3D model of lamprey ER, we inserted E2 into lamprey ER, by overlapping lamprey ER with human ERα. E2 was extracted from human ERα and inserted into lamprey ER using the Biopolymer option in Insight II. Builder from Insight II was used to add the 15α-hydroxyl group to E2 for analysis in lamprey ER and human ERα.

We refined the structure of lamprey ER with E2 and 15α-OH-E2 and human ERα with 15α-OH-E2 using Discover 3 in Insight II. For this energy minimization step, Discover 3 was run for 10,000 iterations, using a distant dependent dielectric constant of 2.

## Results

Figure 3 shows that our 3D model of lamprey ER and the crystal structure of human ERα overlap nicely. The root mean square deviation [RMSD] of their Cα chains is 1.4 Å. In Figure 4A and 4B, we show the interaction of E2 with eight residues from human ERα and lamprey ER. Previous analyses have shown that these residues stabilize E2 in human ER [18]–[20]. Three of these amino acids, Arg-394, Glu-353 and Phe-404 in human ERα, correspond to functionally important residues in the PR [21], GR [22], AR [23] and MR [24], [25]. These steroid receptors contain corresponding arginine and phenylalanine residues, and a glutamine, which is a conservative replacement of glutamic acid.

**Figure 3:** Overlap of 3D model of lamprey ER with human ERα. The 3D model of lamprey ER with estradiol was superimposed on human ERα. There is excellent overlap. The root mean square deviation between the Cα backbone of human ERα and lamprey ER is 1.4 Å.

**Figure 4:** Interaction of E2 with human ERα and the 3D model lamprey ER. A. Interaction between E2 and human ERα. B. Interaction between E2 and the 3D model of lamprey ER. Lamprey ER has stabilizing interactions with the A ring of E2 similar to those in human ERα. His-509 has rotated and does not have a hydrogen bond with the C17-hydroxyl on E2. Instead, Cδ2 has a van der Waals contact with the C17-hydroxyl on E2. Also, Cε and Sδ on Met-409 have stabilizing contacts with C15 on E2.

We selected His-524 because it has a hydrogen bond with the 17β-hydroxyl on the D ring of E2. This hydrogen bond between a substituent on the D ring in E2 and human ERα is not found in other adrenal and sex steroid receptors [21]–[25]. Met-343 and Leu-525 also stabilize the 17β-hydroxyl on E2. Met-421 and Ile-424 have contacts with the 15α-hydroxyl on 15α-OH-E2. We also show an important stabilizing interaction between the backbone oxygen of Glu-419 and His-524 [20].

### Comparison of estradiol binding to human ERα and lamprey ER

As shown in Figure 4A, human ERα has stabilizing hydrogen bonds with the A ring of E2. The phenolic hydroxyl on E2 is 2.8 Å from Oε2 on Glu-353 and 2.9 Å from Nη2 on Arg-394. The side chain on Arg-394 is stabilized further through a hydrogen bond between Nε and the backbone oxygen on Phe-404. Cε2 on Phe-404 also has a stabilizing van der Waals contact with C10 on estradiol.

Figure 4B shows that lamprey ER has similar stabilizing hydrogen bonds with the A ring of E2 as found with human ERα. The C3-hydroxyl on E2 is 2.6 Å from Oε2 on Glu-338 and 3.2 Å from Nη2 on Arg-379. Nε on Arg-379 is 3 Å from the backbone oxygen on Phe-389. Cε2 on Phe-389 has a van der Waals contact with C5 on E2.

Comparison of Figure 4A and 4B reveals significant differences in the interaction between the D ring of E2 and human ERα and lamprey ER. In human ERα, Nδ1 on His-524 is 2.8 Å from the 17β-hydroxyl on the D ring of E2. In addition to this conserved hydrogen bond between His-524 and E2, Cε1 on His-524 has a van der Waals contact with the 17β-hydroxyl, which is 3.4 Å from Cε1. His-524 is stabilized by an interaction with the backbone oxygen on Glu-419, which is 3.3 Å from Nε2 on His-524 [Figure 4A]. The 17β hydroxyl on E2 is 3.8 Å from Sδ of Met-353 and 3.5 Å from Cδ1 of Leu-525. These interactions also stabilize E2 in ERα.

Figure 4B shows that in lamprey ER, His-509 has rotated so that Nε2 is 4.6 Å from the 17β-hydroxyl on E2, which is too distant for a hydrogen bond. As a result of this rotation, Cδ2 on His-509 has van der Waal contacts with the 17β-hydroxyl, C17 and C16 on E2, which are 3.6 Å, 3.9 Å and 3.5 Å distant, respectively, from Cδ2. The 17β-hydroxyl on E2 is 4.4 Å from Sδ on Met-328 and 3.4 Å and 3.5 Å, respectively, from Cβ and Cδ1on Leu-510. The backbone oxygen of Glu-404 is 3.9 Å from Nδ1 on His-509. These distances between lamprey ER and E2 are not as favorable for stabilizing E2 binding as found in human ERα. There are, however, other unique stabilizing contacts between Met-409 on lamprey ER and C15 on E2, which could compensate for the loss of the hydrogen bond between His-509 and the 17β-hydroxyl on E2. Sδ and Cε on Met-409 are 3.7 Å and 3.8 Å, respectively from C15 on E2. For comparison, in human ERα, Cδ1on Ile-424 is 4.07 Å from C15.

### Comparison of 15α-hydroxy-estradiol binding to human ERα and lamprey ER

Figure 5A shows that the stabilizing interactions between 15α-OH-E2 and human ERα are similar to that shown in Figure 4A for E2 and human ERα. However, as found for E2 binding to human ERα and lamprey ER, there are important differences in the interaction between the D ring of 15α-OH-E2 and human ERα [Figure 5A] and lamprey ER [Figure 5B]. The 17β-hydroxyl on E2 still has favorable interactions with His-524, Met-343 and Leu-525 in human ERα. Also, Cε on Met-421 and Cγ2 on Ile-524 are 3.8 Å and 3.2 Å, respectively, from the 15α-hydroxyl on 15α-OH-E2. The backbone oxygen on Glu-419 is 3 Å from Nε2 of His-524, which stabilizes His-524.

**Figure 5:** Interaction of 15α-OH-E2 with human ERα and the 3D model lamprey ER. A. In human ERα, Cγ2 on Ile-424 and Cε on Met-421 have van der Waals contacts with 15α-OH-E2. B. Lamprey ER has stabilizing interactions with the A ring of 15α-OH-E2 that are similar to those in human ERα. His-509 has rotated and does not form a hydrogen bond with the C17-hydroxyl on E2. Cδ2 on His-509 has a van der Waals contact with the C17-hydroxyl. Sδ on Met-406 and Met-409 stabilize 15α-OH-E2.

The 3D model of lamprey ER with 15α-OH-E2 reveals that His-509 and Met-328 do not have the same stabilizing interactions found in the corresponding residues in 3D model of human ERα with 15α-OH-E2. As shown in Figure 5B, in lamprey ER, Nε2 on His-509 and Sδ on Met-328 are 4.5 Å and 5.0 Å, respectively from the 17β-hydroxyl on 15α-OH-E2. These distances are too far for the formation of a hydrogen bond. There are, however, van der Waals contacts between His-509 and the D ring on 15α-OH-E2. Thus, Cδ2 on His-509 is 3.6 Å, 3.9 Å and 3.5 Å from the 17β-hydroxyl, C17 and C16, respectively. Leu-510 still stabilizes the 17β-hydroxyl on 15α-OH-E2. Cβ and Cδ1 on Leu-510 are 3.6 Å from the C17-hydroxyl on 15α-OH-E2. The backbone oxygen of Glu-404 is 3.6 Å from Nε2 on His-509. There also are unique stabilizing contacts between the 15α-hydroxyl on 15α-OH-E2 and Met-406 and Met-409. Cε and Sδ on Met 406 and Sδ on Met-409 are 3.6 Å, 3.5 Å and 2.9 Å, respectively, from the C15 hydroxyl on 15α-OH-E2.

### Met-409 lamprey ER is unique among vertebrate ERs

A BLAST search of GenBank, which contains over 500 ERs from a variety of vertebrates, found that almost all ERs contain an isoleucine corresponding Ile-424 found in human ERα and ERβ [Figure 2]. There were no vertebrate ERs with a methionine at this position.

Interestingly, at this position in ERβ, there is a valine, instead of an isoleucine, in five New World monkeys: *Cebus apella* (brown capuchin) [GenBank: **ABY64736**], *Callithrix jacchus* (white-tufted-ear marmoset) [GenBank: **Q95171**], *Ateles paniscus* (black spider monkey) [GenBank: **ABY64735**], *Pithecia pithecia* (white-faced saki) [GenBank: **ABY64737**], *Callicebus donacophilus* (Bolivian titi) [GenBank: **ABY64738**] and a fish *Acipenser schrenckii* (Amur sturgeon) [GenBank: **BAG82652**] [26]. Valine is a conservative replacement of isoleucine. ERα in the above vertebrates contains the conserved isoleucine.

## Discussion

We have constructed a 3D model of lamprey ER using the crystal structure of human ERα as a template. There is excellent conservation in the structures of human ERα and our 3D model of lamprey ER, as seen in the RMSD of 1.4 Å between their Cα chains [Figure 3].

Comparison of lamprey ER and human ERα in Figures 4 and 5 reveals a conservation of interactions of the A ring of E2 and 15α-OH-E2 with lamprey ER and human ER. It is in the interaction of human ERα and lamprey ER with the D ring on E2 and 15α-OH-E2 that we find a key difference. There is a unique hydrogen bond between Sδ on Met-409 in lamprey ER and 15α-hydroxyl on 15α-OH-E2 [Figure 5B]. In contrast, Ile-524 in human ERα has a van der Waals contact with the 15α-hydroxyl group [Figure 5A]. In lamprey ER, His-509 does not have a stabilizing hydrogen bond with the 17β-hydroxyl on E2 or 15α-OH-E2. There are, however, van der Waals contacts between Cδ2 on His-509 and the D ring of E2 and 15α-OH-E2 [Figure 5B]. These van der Waals contacts and the unique interaction between Sδ on Met-409 and E2 and 15α-OH-E2 appear to compensate for the loss of the hydrogen bond between His-509 and the 17β-hydroxyl on E2 and 15α-OH-E2 [Figures 4B and 5B]. These additional stabilizing interactions may explain the data of Paris et al [10], who found that lamprey ER is activated by E2.

BLAST analysis of GenBank did not find any other ERs with a methionine at the position corresponding to Ile-424 in human ERα. The uniqueness of Met-409 in lamprey ER and the strong conservation of Ile at the corresponding position in human ERα and ERβ and in almost all other ERs in GenBank suggest a functional role for Met-409 in lamprey ER and Ile-424 in human ERα and the corresponding isoleucine in other ERs.

Interestingly, ERβ in five New World monkeys and a sturgeon have a valine instead of isoleucine at the position corresponding to Ile-424 in human ERα. Valine is a conservative replacement of Ile and would have similar van der Waals contacts with 15α-OH-E2, in contrast to the hydrogen bond between Sδ on Met-409 in lamprey ER and 15α-OH-E2. The strong conservation of isoleucine at this position in vertebrate ERα and ERβ suggests that replacement of isoleucine by valine in some New World primates and in a sturgeon may be functionally important.

### Evolutionary Implications

Due to the location of lamprey at the base of the vertebrate line, lamprey is of much interest for understanding the evolution of the vertebrate endocrine system and early events in the evolution of steroid hormone signaling [4], [6], [8], [27], [28]. An important advance towards this goal was the cloning of lamprey ER and the finding that it had strong sequence similarity to human ERα [7]. Our finding that there is excellent conservation of most of the interactions between E2 and amino acids in the steroid-binding pocket in the 3D model of lamprey ER and human ERα [Figure 4] is consistent with the recent report by Paris et al [10] that E2 binding to lamprey ER regulates gene transcription. In this regard, lamprey ER differs from amphioxus ER, which is the most basal chordate with an ER that is clearly orthologous to vertebrate ERs. Unexpectedly, amphioxus ER does not bind either E2 or other common steroids [10], [29] despite the presence of steroidogenic enzymes and E2 in amphioxus [30], [31]. Instead, another nuclear receptor, amphioxus steroid receptor (SR) is activated by estradiol [29]. The evidence for estradiol signaling in amphioxus and the transcriptional activation of lamprey ER by estradiol support earlier proposals that adrenal and sex steroid signaling evolved after the separation of protostomes and deuterostomes [4], [6], [27], [28].

### Environmental implications

Sea lamprey is a pest in the Great Lakes, where lamprey consumes trout and other valuable fish. Our 3D model of lamprey ER identifies a unique structure that interacts with the D ring on E2. This difference from other vertebrate ERs could be exploited to find compounds that selectively inhibit lamprey ER by virtual screening of chemical libraries for binding to our 3D model of lamprey ER. Such contraceptives would provide a means to control sea lamprey.
